# Dose-Dependent Variation in Anticancer Activity of Hexane and Chloroform Extracts of Field Horsetail Plant on Human Hepatocarcinoma Cells

**DOI:** 10.1155/2022/5778411

**Published:** 2022-06-25

**Authors:** Hadeel A. Almasoud, Daoud Ali, Khadijah N. Yaseen, Hanouf Almukhlafi, Norah S. Alothman, Bader Almutairi, Rafa Almeer, Nouf Alyami, Saad Alkahtani, Saud Alarifi

**Affiliations:** Department of Zoology, College of Science, King Saud University, P. O. Box 2455, Riyadh 11451, Saudi Arabia

## Abstract

Horsetail fern plant is botanically known as Equisetum arvense L., and it is a good source of phenolic flavonoids, phenolic acids, and compounds. Anticancer properties of hexane and chloroform extracts of the horsetail fern plant and their mechanisms involved in the anticancer activity on human hepatocarcinoma (HuH-7) cells were examined. Cytotoxicity was evaluated by using MTT (3-(4,5-dimethylthiazol-2-yl)-2,5-diphenyltetrazolium bromide) and NRU (neutral red uptake) assays. Other parameters such as oxidative stress and apoptosis in pretreated hexane and chloroform extracts of the horsetail fern plant were examined in HuH-7 cells. The observation showed that hexane and chloroform extract of the horsetail fern plant exhibited cytotoxicity against HuH-7 cells. The value of IC_50_-24 h of hexane and chloroform extract of the horsetail fern plant was determined as 199.0 *μ*g/ml and 161.90 0 *μ*g/ml for HuH-7 cells, respectively, and on the basis of IC_50_ value, three acute concentrations, viz., 75% of IC_50_, 50% of IC_50_, and 25% of IC_50_, were determined for further study. The lower dose of extracts hexane and chloroform extract of the horsetail fern plant did not show significant toxicity. Higher concentrations of extract induced significant antioxidant effects as well as apoptosis effects. However, exposure to hexane and chloroform extract of the horsetail fern plant upregulated the expression of Bax and p53 in HuH-7 cells. These data suggest that hexane and chloroform extract of the horsetail fern plant plays a significant role in the induction of toxicity via the regulation of oxidative stress in HuH-7 cells. This work may be useful for cancer chemotherapy.

## 1. Introduction

Cancer is one of the most dreadful diseases globally, and it appears to be due to extreme free radical damage, which eventually causes damage to the DNA, lipids, and protein. The horsetail plant scientifically called as *Equisetum arvense* L. (belongs to the Equisetaceae family) is a perennial fern (Figure 1). The horsetail plant has a green-branched sterile stem and grows during the late autumn seasons [1]. The horsetail plant has a medicinal value which was described in European Pharmacopoeia [1]. Extract of the horsetail plant has a gorgeous source of flavonoids, phenolic compounds, and phenolic acid with reducing and antioxidant properties [2, 3] have reported that some Chinese medicinal plant extract was able to detect immunological disorder during tumor disease. Some researchers had reported antioxidant, antifungal, anti-inflammatory, and neuro- and cardio-protective of horsetail plant [4].

A high concentration of extract horsetail plant had induced apoptosis and preoxidant and reduced secretion of IL-6 enzymes [4]. We experimented to confirm the toxicity of extracts of *Equisetum arvense* L. on HuH-7 cells. Aljarba et al. [5] reported that isolated alkaloid and sterol compounds of different medicinal plants induced synergistic anticancer effect on young Swiss albino mice. Reactive oxygen species (ROS) produced by mitochondria not only takes part in signaling of stress in normal cells but also contributes to the initiation of nuclear or mitochondrial DNA mutations that promote neoplastic transformation. Damaging of DNA generates activation of arrest cell growth, and the p53 gene stimulates apoptosis, as per the level of the ratio of oxidative stress [6]). Excessive production of ROS in cells leads to degeneration of mitochondrial membrane potential [7, 8]. have reported that induction of apoptosis is correlated with the generation of ROS. Hegedűs et al., [1] have reported that extract of horsetail plant has shown a preventive effect on oxidative stress and cardiovascular disease in diabetic rats. To my knowledge, there are no studies that have been reported on the toxic nature of hexane and chloroform extracts of the *E. arvense* on HuH-7 cells. In this study, we determined the role of oxidative stress in the toxicity of hexane and chloroform extracts of the *E. arvense* on HuH-7 cells.

## 2. Materials and Methods

### 2.1. Chemical and Reagents

MTT [3-(4, 5-dimethylthiazol-2-yl)-2, 5-diphenyltetrazolium bromide], H2-DCFH-DA), DMSO, Annexin V FITC, and PI dye were bought from Sigma-Aldrich (St. Louis, Missouri, United States). DMEM, fetal bovine serum (FBS), and antibiotics were bought from Gibco, USA.

### 2.2. Plant Material Collection and Preparation of Plant Extracts

In this study, we used *E. arvense*, and it was purchased from the local market in Riyadh, Saudi Arabia (Figures 1(a)–1(c)). The plant was identified by Dr. Jacob Thomas, Taxonomist, Department of Botany and Microbiology at King Saud University, Riyadh, Saudi Arabia. The leaves and stems of the plant have been dried and ground using an electric mill. The plant powder (50 g) was weighed and then placed in a thimble in the Soxhlet extraction apparatus. The extraction process was performed for 24 h using two types of different solvents such as hexane and chloroform [9, 10] ) to obtain the most significant number of secondary metabolic compounds in the plant. The extracts were collected, centrifuged at 5000 rpm for 10 min, and concentrated using a rotary evaporator (Heidolph, Germany) at 45°C. The concentrated extracts were stored in glass vials at 4°C until use. All extracts were dissolved in dimethyl sulfoxide (DMSO) (Sigma) at 50 mg/ml stock (European Medicines Agency, 2016).

### 2.3. Cell Culture and Plant Extract Exposure

Human hepatocarcinoma (HuH-7) cells were bought from American Type Culture Collection (ATCC), USA. HuH-7cells were subcultured in DMEM with 10% FBS and 10000 U/ml antibiotics at 5% CO_2_ incubator at 37°C.

HuH-7 cells were subcultured for 24 h before treatment with hexane and chloroform extracts of the *E. arvense*. Stock solution of extract was prepared in DMSO at 50 mg extract/ml DMSO and diluted according to the experimental concentration (0-200 *μ*g/ml).

### 2.4. MTT Assay

Cytotoxicity of HuH-7 cells due to coexposure of hexane and chloroform extracts of the E. arvense was performed by using the MTT test [11]). In brief, HuH-7 cells (2 × 10^4^) were seeded/well in 96-well plates and kept in the 5% CO_2_ incubator for 24 h at 37°C before experiments for the proper growth of the cells. After incubation, the cells were exposed to various concentrations of hexane and chloroform extracts of the E. arvense (0, 20, 50, 100, 150, 200, and 500 *μ*g/ml) and incubated in a CO_2_ incubator at 37°C for 24 h. At exposure, the culture medium was replaced with a new medium containing MTT solution (0.5 mg/ml) and incubated for 4 hours at in a CO_2_ incubator at 37°C. The produced formazan crystals were dissolved in dimethyl sulfoxide. Then, the plate was read at 570 nm using a multiwell microplate reader (Synergy Fluostar, Germany). Untreated cell set was under identical conditions and served as controls.

### 2.5. NRU Assay

The NRU (neutral red uptake) test was done to quantify the viability of cells (Borenfreund and Puerner, [12]). In brief, HuH-7 cells (2 × 10^4^) were seeded per well in 96-well plates and kept in the 5% CO_2_ incubator for 24 h at 37°C before experiments for the proper growth of the cells. After incubation, HuH-7 cells were treated with a concentration of hexane and chloroform extracts of the E. arvense (0, 20, 50, 100, 150, and 200 *μ*g/ml), and the exposed culture plate was incubated in a CO_2_ incubator at 37°C for 24 h. After incubation, the cells were allowed to incubate for 3 h in a complete medium containing neutral red dye (50 *μ*g/ml). Thereafter, the cells were washed with a washing solution to remove the excess dye. To extract the neutral red dye, a mixture of ethanol (50%) and acetic acid (1%) was filled into each well and kept for 20 min on a shaker. The absorbance was measured at 540 nm by using a multiwell microplate reader (Synergy Fluostar, Germany). Untreated cell set was under identical conditions and served as controls.

### 2.6. Determination of IC_50_ Value 24 h for Extracts of the E. Arvense

The effect of the hexane and chloroform extracts of the E. arvense on cells was measured by counting viable cells by calculating the concentration that inhibits 50% of cell line growth (IC_50_) determined by the dose-response curve graph using the program (OrigenPro 8.5) after repeating the experiment three times [13]).

### 2.7. LDH Assay

Cytotoxicity induced by hexane and chloroform extracts of the E. arvense was assessed by lactate dehydrogenase (LDH) leakage into the culture medium as per LDH cytotoxicity assay kit (Cayman chemical 601170 kit). Briefly, HuH-7 cells were seeded in 96-wells with 100 *μ*l of culture medium for 24 h. Then, the culture medium was removed, and the plant extracts were added (per well) with 200 *μ*l of medium, and 200 *μ*l of medium only (without cells) was added to the three wells (background control), and 20 *μ*g/ml of 10% Triton X-100 solution was added to the three wells (total release), and 20 *μ*g/ml of assay buffer was added to the three wells (Spontaneous release) for 24 h. After incubation, they were centrifuged at 1000 rpm for 5 min. 100 *μ*l of cell supernatant was transferred to a new 96-well plate, and a reaction solution was added 100 *μ*l to each well. The plates were incubated with gentle shaking on an orbital shaker for 30 min at 37°C. Absorbance was read at 490 nm with a plate reader (Synergy Fluostar, Germany).

### 2.8. Catalase Activity

Measurement of catalase activity was based on the peroxidative function of catalase. Briefly, the cells were collected and sonicated in buffer (50 mM potassium phosphate, pH 7.0, containing 1 mM EDTA) followed by centrifugation at 10,000 × *g* for 15 min at 4°C. The supernatant was then assayed for catalase activity using the manufacturer's protocol, and absorbance was monitored at 540 nm by using a plate reader (Synergy Fluostar, Germany). The activity was represented as n mole/(min ml).

### 2.9. Superoxide Dismutase (SOD) Activity

SOD estimation was done in cells collected by centrifugation at 1000 × *g* for 10 min at 4°C. Cell pellets were lysed in cold 20 mM HEPES buffer, pH 7.2, containing 1 mM ethylene glycol tetra-acetic acid, 210 mM mannitol, and 70 mM sucrose. The cells were then centrifuged at 1500 × *g* for 5 min at 4°C. Cell extracts were finally incubated with xanthine oxidase for 20 min according to the manufacturer's protocol, and absorbance of the reaction mixture was measured at 450 nm by using a plate reader (Synergy Fluostar, Germany).

### 2.10. Western Blotting

For western blotting, 20 mg of protein was applied to the lanes of 4% to 12% Bis-Tris Gels (Life Technologies), then blotted onto Immobilon-P membranes (Millipore, Bedford, MA, USA), and incubated with the relevant primary antibodies such as anti-Bax antibody [E63] ab32503 and anti-caspase-3 antibody [E87] ab197202 (Abcam, Cambridge CB2 0AX UK). Appropriate species-specific conjugated secondary antibody goat anti-rabbit HRP (ab205718) was commercially obtained (Abcam, Cambridge CB2 0AX UK). Proteins were detected using the ECL prime kit or the ECL kit (GE Healthcare Tokyo Japan) with an Image Quant LAS 4000 system (GE Healthcare). All protein expression levels were normalized to the levels of GPDH protein expression in each band.

### 2.11. RNA Extraction, cDNA Synthesis, and Real-Time PCR

The RNA was reverse-transcribed using RT-PCR kits (Applied Biosystems, Foster City, CA, United States) with an oligo d (T) 16 primer under standard conditions. Real-time PCR amplification was performed using a Light Cycler 480 (Roche, Basel, Switzerland) and 2 *μ*l of purified cDNA product, 5 *μ*l of sense primer (10 pmol/ml), 5 *μ*l of antisense primer (10 pmol/ml), 1 ml of Light Cycler Fast Start DNA Master SYBR Green I (Roche), and 0.8 ml of MgCl2 (25 mmol/L). Commercial glyceraldehyde phosphate dehydrogenase (GAPDH) primer sets were used for PCR amplification under the conditions recommended by the manufacturer (Table 1). GAPDH served as an internal reference gene, and the relative change was calculated by relative quantification, applying the formula by the 2−△△Ct method.

### 2.12. Statistical Analysis

Statistical analysis was performed using SPSS software (Ver.22; SPSS Inc., Chicago, IL, USA). Data were examined using one-way ANOVA, followed by a post hoc LSD (least significant difference) test, and the results were presented as average ± SE. *p* value < 0.05 was considered statistically significant.

## 3. Results

### 3.1. IC_50_ Value 24 h

The IC_50_ was determined by the dose-response curve graph using the program (OrigenPro 8.5) (Figures 2(a) and 2(b)), and it was determined based on the MTT test result. We observed the IC_50_ value of 24 h 199 *μ*g/ml for hexane and 161 *μ*g/ml for chloroform extracts of the *E. arvense* (Figures 2(a) and 2(b)).

### 3.2. Cytotoxicity

The cell viability of HuH-7 cell lines was reduced significantly in a dose-dependent manner due to hexane and chloroform extracts of the *E. arvense* exposure (Figures 3(a) and 3(b)). The viability of HuH-7 cell line was decreased to 83%,84%, 65%, 62%, 53%, and 13% for hexane plant extract and 88%, 66%, 57%, 55%, 46%, and 14% for chloroform plant extract in 24 h at all concentration (20 *μ*g/ml, 50 *μ*g/ml, 100 *μ*g/ml, 150 *μ*g/ml, 200 *μ*g/ml, and 500 *μ*g/ml), respectively, through MTT test (Figure 3(a)).

The viability of HuH-7 cell line was decreased in all concentrations to 86%, 78%, 73%, 61%, and 55%, respectively, for hexane plant extract, and 88%, 83%, 66%, 49%, and 46%, respectively, for chloroform plant extract in 24 h through NRU test (Figure 3(b)).

Furthermore, the results showed that plant extract reduced viability for both solvents with significant differences (Figures 3(a) and 3(b)).

The LDH test results indicate that compared to control, the loss of membrane integrity was slightly increased to 104%, 107%, and 114% for hexane plant extract and to 116%, 126%, and 132% for chloroform plant extract in 24 h (control, 25, 50, and 75% of the IC_50_, respectively) (Figure 4).

### 3.3. Oxidative Stress

HuH-7 cell lines were exposed with *E. arvense* extract (25%, 50%, and 75% of the IC_50_ value in *μ*g/ml) for 24 h, and CAT and SOD enzyme activity was measured. The results showed that CAT activity was increased maximum at lower concentrations (25% of the IC_50_ value) for chloroform *E. arvense* extract, and it was decreased at higher concentrations (50% and 75% of the IC_50_ value) for hexane and chloroform *E. arvense* extract (Figure 5(a)). SOD enzyme was increased at lower concentration (25% of the IC_50_ value) and decreased at higher concentration (50% and 75% of the IC_50_ value) for hexane and chloroform *E. arvense* extract (Figure 5(b)). The results showed that compared to control, the E. arvense extracts induced CAT and SOD activity in a dose-dependent manner (Figures 5(a) and 5(b)).

### 3.4. Immunoblotting

To confirm the apoptosis due to the effects of plant extract (25%, 50%, and 75% of the IC_50_ value in *μ*g/ml) for 24 h, on HuH-7 cells, we have determined the expression of the apoptotic protein in cells after exposure to hexane and chloroform *E. arvense* extract. In HuH-7 cell line, the result showed that caspase-3 protein expression was upregulated at all concertation to 1.3, 1.3, and 1.4, respectively, for hexane plant extract and more upregulated to 2.8, and then, it was downregulated to 2.2 and 1.7, respectively, after treating with chloroform plant extract (Figures 6(a) and 6(b)).

While the result showed that Bax protein expression was upregulated at all concentrations (1.1, 1.4, and 1.3, respectively), for hexane plant extract and upregulated at the concentration 1.1 and 1.5, then it was downregulated to 0.9 after being treated with chloroform plant extract (Figures 6(a) and 6(b)).

### 3.5. Apoptotic Gene Expression

To examine the expression level of the apoptotic genes in human liver cell lines, RT-PCR analysis was performed. In HuH-7 cell line, the result showed that p53, caspase-3, and Bax mRNA expression compared to control were increased at all concentrations to 5.4, 6.4, and 7.1, 3.7, 3.8, and 2.2, and 1.5, 3.0, and 2.7, respectively, for hexane plant extract and to 2.3, 3.0, and 3.6, 2.5, 3.0, and 3.4, and 1.9, 2.0, and 1.3, respectively, for chloroform plant extract. On the other hand, the Bcl-2 mRNA expression was decreased at all concertation to 0.9, 0.6, and 0.3, respectively, for hexane plant extract and to 0.8, 0.6, and 0.3, respectively, for chloroform plant extract (Figures 7(a) and 7(b)).

## 4. Discussion

Several reports and studies have indicated that cancer is a major cause of death worldwide, causing nearly 10 million deaths, and liver cancer was the most common cause of death with 830,000 cases (WHO, 2020). We used extracts of *E. arvense*, which is considered one of the medicinal plants that current research has confirmed to have many pharmacological applications, and peer-reviewed studies showed that these pharmacological activities of medicinal plants are due to their valuable chemical components, which mainly include alkaloids, triterpenoids, flavonoids, phenols, and tannins [14]. In a previous study, *E. arvense* did not show any noticeable toxic effects; however, clinical trials are necessary (Kotwal [15]. In other studies, the extract of *E. arvense* inhibited the proliferation of cancer cells and extended the lifespan of mice [16]).

So, researchers are keen to investigate the underlying mechanism of toxicity of hexane and chloroform extracts of the E. arvense exposure on HuH-7 cells. In the present experiment, exposure of hexane and chloroform extracts of the *E. arvense* to cells for 24 h demonstrated significant cytotoxicity and apoptotic effects on hepatic cancer cells. In addition, a significant decrease in SOD and increase in catalase enzyme at lower concertation were observed. A recent study done by Zalewska et al. [17] showed that cancer cells mostly contain few antioxidant enzymes such as CAT, GSH-PX, and SOD, which play a dynamic role in cellular protection against ROS in normal cells. Increasing of oxidizing agents such as ROS affects cell organelles and cellular compounds, such as carbohydrates, lipids, proteins, and DNA molecules [18]), and the cells respond through protective enzymatic defense mechanisms such as CAT and SOD to reduce harmful ROS production. Moreover, it has been reported that low expression of SOD correlates with hepatocellular carcinoma mortality [19]). Also, cell death by apoptosis acts as a barrier to the development of cancer [20]. The extracts of *E. arvense* induced apoptosis of HuH-7 cell lines in a dose-dependent manner, and we found that the gene expression level of caspase-3, Bax, and p53 were increased, in contrast to the same doses which lowered the level of bcl-2. The Bax has been shown to be regulated by p53 and to restrict tumorigenesis, and it is essential for apoptosis, while Bcl-2 binds and inhibits the activity of Bax and proapoptotic proteins, thus preventing apoptosis [21]. Taken together, upregulation of p53 leads to activation of proapoptotic members of the Bcl-2 family, such as Bax, and induces permeabilization of the outer mitochondrial membrane, which releases soluble proteins from the intermembrane space into the cytosol, where they promote caspase-9 activation and which further activates caspase-3, which lead to apoptosis [22, 23].

## 5. Conclusion

The current finding provides evidence for the potential efficacy of *E. arvense* extracts, and the results obtained in this work indicate that this extract may be useful as an anticancer drug by activating antioxidant enzymes and programmed cell death pathways. However, there is a need for further investigation using different molecular tests *in vivo* models.

## Figures and Tables

**Figure 1:** (a–c) *Equisetum arvense.*

**Figure 2:** Determination of IC_50_ value-24 h of (a) hexane and (b) chloroform extracts of E. arvense for HuH-7 cells.

**Figure 3:** Hexane and chloroform of plant extracts of *E. arvense* induced cytotoxicity on HuH-7 cell line in a dose-dependent manner for 24 h: (a) MTT assay and (b) NRU assay. Each value represents means of three experiment. *p* value < 0.05 vs. control.

**Figure 4:** Hexane and chloroform of plant extracts of *E. arvense* induced cytotoxicity on HuH-7 cell line in a dose-dependent manner for 24 h. Each value represents means of three experiment. *p* value < 0.05 vs. control.

**Figure 5:** Hexane and chloroform of plant extracts of *E. arvense* decreased oxidative stress biomarkers in HuH-7 cell line for 24 h: (a) catalase level and (b) SOD level in cells. Each value represents means of three experiment. *p* value < 0.05 vs. control.

**Figure 6:** Western blotting of protein involved in apoptosis: (a) Bax and caspase-3 expression level in cells. (b) Relative quantification of protein expression level. GPDH was used as internal control to normalize the data. Each value represents means of three experiment. *p* value < 0.05 vs. control.

**Figure 7:** Expression of apoptotic gene in (a) hexane and (b) chloroform of exposure of plant extracts of *E. arvense* in HuH-7 cell line for 24 h. Each value represents means of three experiment. *p* value < 0.05 vs. control.

**Table 1:** The sequences of primers.

Gene	Primer F sequence (59->39)	Primer R sequence (5,->39)	Product size
*β-Actin*	5′-CACCATTGGCAATGAGCGGTTC-3′	5′-AGGTCTTTGCGGATGTCCACGT-3	131 bp
*Caspase-3*	5′-TGTTTGTGTGCTTCTGAGCC-3′	5′-CACGCCATGTCATCATCAAC-3	123 bp
*Bax*	5-ATGTTTTCTGACGGCAACTTC-3′	5′-AGTCCAATGTCCAGCCCAT-3	82 bp
*Bcl-2*	5-ATGTGTGTGGAGACCGTCAA-3	5-GCCGTACAGTTCCACAAAGG-3′	142 bp
*P53*	5′-AGAGTCTATAGGCCCACCCC-3′	5′-GCTCGACGCTAGGATCTGAC-3	81 bp

## Data Availability

The original contributions presented in the study are included in the article; further inquiries can be directed to the corresponding author.
